The article "Design of Association Application System of Face Recognition and Test-Tube Barcode Based on CNN" was published in 2022. Journal: Comput Math Methods Med.

# Design of Association Application System of Face Recognition and Test-Tube Barcode Based on CNN

**DOI:** 10.1155/2022/1987857

**Published:** 2022-08-24

**Authors:** Zhangning Zhou, He Shi, Xuemin Niu

**Affiliations:** ^1^General Practice Department, Huzhou Central Hospital, Huzhou 313003, China; ^2^Affiliated Central Hospital Huzhou University, Huzhou 313000, China; ^3^Zhejiang Health Technology Co., Ltd., Hangzhou 311100, China; ^4^Clinical Laboratory, Huzhou Central Hospital, Huzhou 313003, China

## Abstract

In order to improve the standardization and accuracy of business process management of laboratory department in hospitals, combined with convolutional neural networks (CNN) and face recognition technology, an association application system of laboratory face recognition and test-tube barcode is designed by inputting patient's face and blood test-tube barcode into the system for storage. When the patient logs into the system again, the system uses the patient's face to automatically search for a matching test-tube barcode to obtain the test results. The simulation results show that the system can accurately recognize the face and match the corresponding test-tube barcode, and the accuracy and ROC of face recognition are 0.85 and 0.94, respectively. In addition, when the patient's face is within 5 m from the system camera, the accuracy of face recognition can reach 100%. It can be seen that the system designed in this paper shows good performance.

## 1. Introduction

With the continuous development of computer vision and image processing technology, face recognition technology began to be applied to many fields, and it gradually becomes a hot topic. At present, many technologies are applied to face recognition, such as Haar feature matching and BP neural network [1–14]. These technologies play an important role in face recognition and detection. In specific studies, Ghazal and Ghazal proposed the Fisherface algorithm, which has attracted more attention [15]. In addition to this method, Abratenko et al. designed Haar-like, which has also achieved certain effects in face recognition scenes [10]. With the application of face recognition in various fields, how to apply it to the medical field has become a hotspot of current research. For example, Lyanpen and others applied face recognition to patient admission management, which greatly saved the time of admission [16]; Mamata and Ninad combined face recognition with voice assistance to help patients call nursing services [17]; Jenifa et al. applied face recognition to patients' expression evaluation, which can assist in the evaluation of patients' emotions [18]. However, it has been found in practice that the application of face recognition technology in medical institutions is increasing, but there are not many studies on the application of bar codes in laboratory departments. Therefore, it is necessary to strengthen the research in this field. It is hoped that through this application, the obstacle between face recognition and test results can be broken through, so that patients can obtain the report results only through the face instead of through the conventional QR code. This is the problem that has not been solved or is trying to be solved in the previous research. With the help of such new technology, the business process of the laboratory can be simplified, so as to improve efficiency and gradually realize the goal of paperless office.

## 2. Face Target Detection Based on SSD

The SSD algorithm is used to realize face detection. The core part of the algorithm is the anchor mechanism, which takes each point as the center point of candidate area and makes regression for location and target category. Moreover, the multiscale feature map is utilized in the detection process, which is helpful to improve the accuracy of detection results. In general, this algorithm belongs to a method based on deep learning, in which there is no need to extract candidate box, the operation is relatively simple, and the application prospect is broad. However, the SSD algorithm also faces some challenges in application, especially for different fields, its requirements for image detection and recognition are different, and its image processing is also different. This research is mainly aimed at patients' face recognition. In the image detection method, the requirement for accuracy is higher. Therefore, in this article, how to use the SSD algorithm to accurately identify patients is an important challenge. SSD is chosen because it is a new convolutional neural network face detection framework. Its face detection mechanism is different from the network using candidate frame mechanism. Different convolution layers of convolution neural network have different receptive fields and different feature dimensions. The receptive fields of shallow neurons are small, the output feature map is large, the receptive fields of deep neurons are large, and the output feature map is small. Therefore, in the SSD convolution network, different levels of feature maps are not only used as the input of the lower convolution layer to extract features but also as the input of the detection and prediction network to output the face category score and accurately locate the face. The basic principle of the algorithm is shown in Figure 1 [19–22].

As can be seen from Figure 1, this algorithm model can be divided into several parts, among which the initial part is VGG16, the backbone networks are VGGNet, Inception, etc. Con4_3 and Conv6 are all convolution layers. Then, the full connection layer is *FC6*, and *FC7* is converted into the convolution layer. In addition, the recognition layer is after Conv7, which requires continuous downsampling until (1 × 1). The structure and function of each layer are different. There is a special classifier layer in Con4_3 layer, through which feature map can be extracted. This convolution layer also exists in other layers, such as Con8_2 and Con11_2. The corresponding feature map can also be extracted.

The extracted feature map is input into the detection layer to obtain location and category information. During this process, default boxes need to be defined to obtain the target offset and category score.

The basic form of loss function is as follows [23–25]:

(1) $$\begin{array}{c} L\left(x,c,l,g\right)=\frac{1}{N}\left(L_{\text{conf}}\left(x,c\right)+\alpha L_{\text{loc}}\left(x,l,g\right)\right), \end{array}$$

where *L*_loc_ and *L*_conf_ are regression and classification loss functions, respectively, and smooth and softmax functions are used for them, respectively. *N* is the number of positive samples in the prediction box, *c* is the category confidence prediction value, *l* is the position prediction value corresponding to the prediction box, *g* is the position marked by GT, and *a* is the weight coefficient of position loss and confidence loss.

In this design, the backbone network is ResNet, and feature learning can be carried out in combination with feature map. However, in order to obtain high-precision detection results, it is generally necessary to use multiple feature maps. For the SSD algorithm, six feature maps can meet the requirements of detection.

## 3. Face Recognition Based on FaceNet

The FaceNet algorithm is used to map images to the multidimensional space, and the similarity of face is calculated and compared. Specifically, face similarity needs to be quantitatively compared according to the size of the spatial distance; that is, the image of a person is generally small in the spatial distance, and the image between different *g* individuals will maintain a high spatial distance. In this way, the detection of the face can be realized, and then the identity of the person is determined.

For the FaceNet algorithm, triplet loss function and image mapping method are adopted in the training process, so as to obtain the corresponding vector space. The specific network structure is shown in Figure 2 [26–28].

As can be seen from Figure 2, batch represents training data, which includes more triples. Then, the process of feature extraction is carried out, and the image transformation and normalization operations are successively carried out; thus, vector embedding can be obtained. Then, it is input into the triplet loss function. On the basis of obtained feedback, the update of embedding is achieved. After completing training, the triplet loss is transformed, and the similarity measurement results are obtained through extracting embedding and calculating Euclidian distance.

In the last part of the FaceNet model, triplet loss function is required to complete the training process, in which the input feature vectors are negative feature vector, positive feature vector, and anchor feature vector. Feature vectors 1 and 3 belong to the different type of samples. Feature vectors 2 and 3 belong to the same type of samples, which needs to perform feature optimization, so as to ensure that the different type of samples can keep a large distance, while the same type of samples has a small distance. Triplet loss is shown as follows:

(2) $$\begin{array}{c} {\left\|f\left(x_{i}^{a}\right)-f\left(x_{i}^{p}\right)\right\|}_{2}^{2}+\alpha <{\left\|f\left(x_{i}^{a}\right)-f\left(x_{i}^{n}\right)\right\|}_{2}^{2}, \end{array}$$

where *f*(*x*_*i*_^*p*^) and *f*(*x*_*i*_^*n*^) represent the different or same types of sample pairs, *f*(*x*_*i*_^*a*^) stands for anchor vector, and *α* stands for interval, which is used to adjust the sample distance.

The basic form of loss function is as follows:

(3) $$\begin{array}{c} L_{i}=\overset{N}{\underset{i}{\sum }}\left[{\left\|f\left(x_{i}^{a}\right)-f\left(x_{i}^{p}\right)\right\|}_{2}^{2}+{\left\|f\left(x_{i}^{a}\right)-f\left(x_{i}^{n}\right)\right\|}_{2}^{2}+\alpha \right], \end{array}$$

where *N* represents the number of sample pairs. Based on this function, sample similarity can be measured, and Euclidean distance is generally adopted in the specific calculation. *L*_*i*_ represents the triplet loss function.

The basic flow of the FaceNet algorithm is shown in Figure 3.

As can be seen from Figure 3, SSD face recognition is divided into two parts. One part is to train the pictures to obtain the trained SSD network, and then the trained network is used to test the pictures, which are compared with the correct face features, so as to judge whether they are the same person. Finally, the purpose of face recognition is achieved.

## 4. Business System Construction of Laboratory Department Based on Face Recognition

### 4.1. Design of Overall System Architecture

The purpose of this paper is to try to apply face recognition to the business of laboratory departments, so that patients can log in system to query test reports through face. Therefore, based on this particular scenario, and combined with the specific business of the laboratory department, the system is divided into several parts, including the client, server, and database part, in which detailed analysis and design are made for each part. The specific architecture is shown in Figure 4.

In Figure 4, http protocol is used for communication between the server and the client. When the client needs to obtain resources from the server, get method can be adopted, and when the client transfers resources to the server, post method can be adopted.

### 4.2. Construction of System Network Architecture

The overall network architecture of system is shown in Figure 5.

In the overall architecture, each system of the hospital is included, which is connected through a unified network, so as to obtain various data of the hospital system and finally achieve the purpose of data sharing of the whole hospital. In other words, face recognition can not only realize the query of report results of inspection department but also lay the foundation for other queries and applications.

### 4.3. Process of Some Functions of the System

#### 4.3.1. Face Swiping Detection Process

The face swiping detection process is shown in Figure 6.

When patients are collecting specimens, they are verified by the face recognition system in the cloud, and the face features are compared with the comparison source through the background. After verification, the results are returned.

#### 4.3.2. Process of “Face Recognition+Preplacement Bar Code”

The identification process is shown in Figure 7.

The detailed steps in Figure 7 are as follows:

- Firstly, carry out the user identity authentication process. In the specimen collection process, set the mode of “face swiping” and then select the face meeting the requirements to realize the identity authentication
- Secondly, set the mode of bar code and check the label of preplacement bar code of disposable vacuum tube using the equipment provided by the manufacturer
- Moreover, select Confirm key. The user's information can be extracted from HIS, and it can be associated with the “pre-placement bar code” test tube
- Finally, upload the obtained results by inspectors

#### 4.3.3. Process of Printing Report by Swiping Face

The process is shown in Figure 8.

As can be seen from the figure, users need to swipe their faces through the self-service machine first and then compare the collected face images. After verifying the user's identity, the corresponding laboratory sheet is queried, and it can be printed out.

## 5. Method and System Verification

### 5.1. Face Detection and Verification Based on SSD

#### 5.1.1. Data Processing of WIDER FACE

The data set of this study is the public wide face dataset. WIDER FACE dataset is utilized to test the designed SSD model, which has rich face samples and is widely used in face recognition and detection [21–25], where it contains a total of 32,203 face images under different conditions such as illumination, occlusion, and scale. This data set is actually extracted from 61 event category videos, which are extracted and divided according to each event category. Thus, there are three parts obtained, which are, respectively, used for training, testing, and crossverification, and the ratio of the three part is 4 : 5 : 1. Partial images of this dataset are shown in Figure 9.

The first is to convert the format of this dataset; thus, PASCAL VOC format is obtained. After the conversion, three directories, namely, annotations, image sets, and JPEG images, are obtained. The information stored in each directory has certain differences, namely, picture interpretation, image collection, and picture.

#### 5.1.2. Face Detection Model Training Based on SSD

TensorFlow is mainly used for training. After the completion of model construction, the code is adjusted according to the requirements of face detection, and then the training process is completed by invoking the relevant interface according to the data set.

After the preprocessing, test.txt and train.txt can be generated, and data sets in PASCAL VOC format are obtained. The create_pascal_tf_Record.py file is then packaged to obtain the TFRecord format and the corresponding file. The specific packaging information involves path, file name, and image size information. Once the information is packed, training can be carried out.

In the training process, the SSD algorithm is mainly adopted, and the model_main.py file is directly utilized in this process, which is located in the source code of the SSD algorithm. After modifying the configuration file and relevant parameters, all can be used in the process of model training.

TensorFlow is used in this experiment. The configuration files of the SSD algorithm model are all located in configs in the sample directory. However, face detection cannot be performed directly in general, so it needs to be modified appropriately, where ssd_resnet50_v1_fpn_shared_box_predictor_640 × 640_COCO14_sync.config is modified as follows:

Here, train.record and test.record are used as training data and test data, respectively. The parameters are set reasonably; that is, image_resizer is 256^∗^256, numclass = 1, batch_size = 24, and num_steps = 100000. In addition, sigmoid and smooth functions are used for classification and regression loss, respectively.

After the configuration file is set, the Python script program is executed in the terminal, and the name of file is model_main.py. And then the relevant interface is called for metatraining, and the formed information is displayed in the terminal. The AP curve of detection is shown in the following Figure 10.

AP values can be obtained, including three IoU ratios, namely, small, medium, and large. Among them, the AP values of large, medium, and small targets are different, which are 0.626, 0.28,7 and 0.038, respectively.

The training set used in the experiment includes CelebA, CASIA-facev5, and CASIA-WebFace, while the test set is LFW dataset.

#### 5.1.3. Model Test

Test the trained model, restore graph in combination with the obtained model file, and then perform the forward calculation process. In addition to this method, graph of the model can be restored first, and then pb files containing network structure and parameters can be generated. On this basis, forward calculation can be performed. The advantage of this method is high efficiency and convenient for system design and testing.

In TensorFlow, the integrated export_inference_graph.py file is used to convert graph to pb files. This file can be called directly from the terminal, and then the conversion can be achieved; thus, the corresponding pb file is obtained. However, the obtained model file at this time cannot be used directly, in which parameters need to be adjusted, and the specific parameter setting is shown as follows: the input_type needs to be set to image_tensor. Then, add the path of ssd_resnet50_v1_fpn_shared_box_predictor_640640_coco14_sync_face.config to this file. After all the information is modified and verified correctly, export_inference_graph.py can be called at the terminal. After parameters such as pb file name and storage path are set well, the corresponding face_detection_model. pb file can be obtained.

It can be seen that a test_model.py script is written to call the previously generated face_detection_model.pb file. After the test set data is input, face detection is carried out, and the detected faces are marked, including certain differences in posture, skin color, and other aspects of a variety of face images.

The final processed results are shown in the following Figure 11.

As can be seen from the test results, the model achieves good results in face detection, realizing multiface detection. In addition to the detection of the positive face, the side and each color of the face can be effectively detected, which has high robustness and is suitable for the design of actual face detection function.

### 5.2. Face Recognition Model Training Based on FaceNet

#### 5.2.1. Data Set Preprocessing

It is necessary to use appropriate data sets during algorithm testing. In this study, multiple data sets are selected, including CelebA, CASIA-faceV5, CASIA-WebFace, and LFW data sets, so as to verify the validity of FaceNet algorithm.

#### 5.2.2. Face Recognition Model Training Based on FaceNet

The train_tripltloss.py script file can be directly used during training, which is located in the FaceNet source code. This file needs to be adjusted according to the requirements of specific applications. Here, epoch_size, batch_size, and max_nrof_epochs are set to 1000, 30, and 500, respectively. At the same time, adjust_brightness and adjust_contrast methods need to be added to improve the robustness of the model. After the modification is complete, enter the four data sets described previously for training.

In the training, the data sets are combined appropriately to verify the training effect of using different data sets, so as to determine the optimal model. Firstly, Celeba_160 and CASIA-WebFace_160 are merged into a new dataset Webface-Celeba_160. Then, start the training process and input the merged data sets and the previous three data sets, respectively, for training. Thus, four models can be obtained. Then, input test set and verify the application effect of each model, and on this basis, it can determine the optimal model. The loss diagram in training is shown as following Figures 12–14.

Through the comparison of loss functions in Figures 12–14, it can be seen that in the identification of FaceNet, the value of loss function in the combined data set is the smallest, indicating that FaceNet is more suitable for the mixed picture data sets.

#### 5.2.3. Model Test

In this test process, the validate_on_lfw.py file is used, and it is also located in the FaceNet source code. The test set is LFW, from which 6000 sample pairs are extracted, specifically divided into positive and negative sample pairs, and the number of the two is 5700 and 300, respectively. Tests are carried out for each training model, and the difference of each model is clarified through ROC diagram analysis. The ROC curve is drawn according to FPR and TPR, while FPR and TPR are calculated as follows [26–28]:

(4) $$\begin{array}{c} \text{FPR}=\frac{\text{FP}}{\text{FP}+\text{TN}}, \end{array}$$

(5) $$\begin{array}{c} \text{TPR}=\frac{\text{TP}}{\text{TP}+\text{FN}}. \end{array}$$

Thus, the optimal model is determined, and the final test results are shown as following Figures 15–17.

As can be seen, the test result accuracy of the model trained by CelebA and CASIA-WebFace data set is high, where accuracy and ROC are higher than 0.85 and 0.94, respectively. In addition, after the training set is merged, the obtained model also can achieve good results in the test, and its accuracy is basically consistent with CelebA and CASIA-WebFace. The model trained based on this data set can be used for face recognition, and it has higher robustness. Therefore, this model is finally selected in this paper.

### 5.3. System Test

#### 5.3.1. Function Test of Face Detection

Tests are carried out under normal lighting conditions to detect the effect of face recognition. During the experiment, face posture and test distance are adjusted to analyze whether the detection effect can be achieved.

There are three testers, all of whom need to be tested 60 times, namely, 15 times for the front and side faces, 15 times for the test distance between 5 m and 10 m, and below 5 m. After the setup is completed, the test is carried out, and the final results are shown in Table 1.

#### 5.3.2. Function Test of Face Recognition

Face recognition is divided into two parts, namely, registration part and login part. During the test, face images are collected from the front, and the distance from the camera is within 5 m. The test is carried out under normal lighting conditions, so as to verify the effect of face recognition and the login time.

There are three testers. Both tester 1 and tester 2 need to register. After registration, the login test will be conducted. Tester 3 performs the login test directly without registration and records the test results. The specific information is shown in the following Table 2.

## 6. Conclusion

In conclusion, the application of face recognition in the laboratory department can effectively improve the recognition accuracy of patients. Through the deep learning algorithm, the recognition accuracy can reach 100% within a distance of less than 5 m, which shows that the application of the deep learning algorithm to the QR code association system of the inspection department has a certain accuracy. At the same time, the identification system can effectively establish the relationship between patients and test results in the test department, so as to greatly improve the information and intelligence level of test department. The innovation of this study is to apply face recognition to the QR code recognition of the laboratory department, so as to connect the patients with the test results of the laboratory department, so that the patients can query the results through face recognition.

However, the focus of this study is only to apply deep learning to face recognition and test tube bar code association system. The main direction of next step of this research should be how to apply deep learning to query the test results.

## Figures and Tables

**Figure 1:** Principle of the SSD model.

**Figure 2:** FaceNet network structure.

**Figure 3:** FaceNet recognition.

**Figure 4:** Design of overall system architecture.

**Figure 5:** Overall architecture of the system.

**Figure 6:** Face swiping detection process.

**Figure 7:** Process of “face recognition+pre-placement bar code.”

**Figure 8:** Process of printing report by swiping face.

**Figure 9:** Partial images in WIDER FACE dataset.

**Figure 10:** AP curve of target detection.

**Figure 11:** Target detection results of SSD.

**Figure 12:** Loss diagram of training set WebFace.

**Figure 13:** Loss diagram of training set CelebA.

**Figure 14:** Loss diagram of training set WebFace-CelebA.

**Figure 15:** ROC diagram of training set WebFace.

**Figure 16:** ROC diagram of training set CelebA.

**Figure 17:** ROC diagram of training set WebFace-CelebA.

**Table 1:** Test table of face detection.

Test project	Distance < 5 m (front face)	5 m < distance < 10 m (front face)	Front face (distance < 5 m)	Side face (distance < 5 m)
Detection rate	100%	86.7%	100%	100%
Average time	398 ms	473 ms	395 ms	414 ms

**Table 2:** Face recognition test table.

Tester	No. 1 (registered)	No. 2 (registered)	No. 3 (unregistered)
Login success rate	100%	100%	0%
Average time	623 ms	618 ms	0 ms

## Data Availability

The experimental data used to support the findings of this study are available from the corresponding author upon request.
